# Surface Defect Detection Method Based on Improved Attention Mechanism and Feature Fusion Model

This article has been retracted.

**DOI:** 10.1155/2022/3188645

**Published:** 2022-03-03

**Authors:** Yongbin Chen, Guitang Wang, Qinshen Fu

**Affiliations:** School of Electromechanical Engineering, Guangdong University of Technology, Guangzhou, Guangdong 510006, China

## Abstract

Cylinder liners are important to automobile engines. The appearance quality will directly affect the life and safety of the engines. At present, the appearance quality inspection of cylinder liners mainly relies on manual visual judgment, which is easily affected by the subjective factors of inspectors. This paper studies improved machine vision to realize surface defect detection. It proposes the improvement of the attention mechanism and a feature fusion method to locate and classify the defect. Experiments show that the method proposed in this paper has improved both accuracy and speed, and it can detect defects in production and realize industrialization. At the same time, the method studied in this paper has the value of popularization and application for appearance defect detection in other fields.

## 1. Introduction

Cylinder liners are important to automobile engines. The appearance quality will directly affect the life and safety of the engines. This paper proposes the improvement of the attention mechanism and a feature fusion method to locate and classify the defect, which has improved both accuracy and speed. The surface defect will indicate that the cylinder liner has a major internal quality problem, which may cause the internal combustion engine to work abnormally and cause safety problems. At present, the inspection of the surface quality of cylinder liners mainly relies on manual inspection methods. Manual inspection methods are unable to meet production requirements, especially for small defects. At the same time, long hours of eye work are harmful to the health of inspectors. Therefore, manual inspection is no longer suitable for the current requirements of large-scale industrial production. Compared with human eyes, computer vision can improve efficiency and accuracy, and it is safe and reliable because of its noncontact type. However, traditional machine vision inspection algorithms are less flexible in feature extraction, and feature extraction algorithms need to be constructed with the types of defects.

Compared with traditional machine vision algorithms, deep learning algorithms not only show higher stability and adaptability when facing changing scenes and targets but also have higher detection accuracy [1]. This paper proposes a deep learning-based defect detection method to realize surface defect detection. The content tested in this paper is the “raised” and “unsintered” surface defects of the nonburr cylinder liner, which are defined as follows:

  Unsintered: the unsintered shape that appears on the surface of the thornless cylinder liner is generally strip-shaped. The length of the defect must not exceed 10 mm and the width must not exceed 5 mm. There are multiple unsintered shapes within the same field of view. The distance must be more than 10 mm, otherwise, no matter how small its size is, it will be regarded as a defect.
  Raised: this type of defect mainly manifests as flat or convex stains. When the diameter exceeds 5 mm, it will be regarded as a defect, and no more than 3 bumps are allowed within the same field of view.

## 2. Related Work

In 2018, Essid et al. [2] used CNN to realize the automatic detection of the metal box surface. Among them, in order to better process data with nonlinearity and sparsity, the autoencoder is used to build a deep neural network structure, and the Gaussian method is used for regression to learn the probability model of the network output result. Compared with the KNN and SVM methods, the false detection rate of this method has decreased.

In 2019, Huang et al. [3] realized the surface quality inspection of engine parts based on the faster R-CNN model. In this method, in order to improve the detection accuracy and detection speed of the model, the structure of ROI pooling is improved, and the detection accuracy is finally increased to 96.8%. In the same year, Ramalingam et al. [4] used a lightweight detection model-SSD MobileNet to detect defects on the surface of the aircraft in order to improve the detection speed of the network. In order to reduce the amount of calculation, the obtained image was scaled and zoomed. The first-level network model-MobileNet v2 [5] builds its detection model and uses feature maps of different scales in the detection network to perform regression prediction, and the final detection accuracy reaches 93.2%.

In 2020, Zhang and Zhang [6] used the deep learning method to detect the surface defects of the cans. First, the corresponding image preprocessing method was used to perform the corresponding cropping, normalization, and other operations on the collected surface images of the cans. Based on the VGG16 network, a defect detection model was designed. After training and optimization, the classification accuracy of the network reached 98.2%.

In 2021, Damacharla et al. [7] used the TLU-Net network to detect steel surface defects. In this research, after studying a series of deep learning models, the detection model framework U-Net [8] is finally determined, and corresponding improvements are made on the basis of U-Net, combined with ResNet [9] and DenseNet [10], to solve the degradation problem of deep networks, the feature extraction ability of the network has been strengthened, and the detection accuracy has been improved by 12%.

## 3. System Architecture

### 3.1. Detection Principle of YOLOv4

In YOLOv4, the main detection steps are completed in the “Prediction” part of Figure 1. As mentioned in the previous algorithms in the YOLO series, the YOLOV4 algorithm also belongs to the anchor-based series. Therefore, it is necessary to use a clustering algorithm on the labeled data to obtain the anchor boxes. The detection is completed on three feature maps of different sizes. Taking the input image of 416 × 416 as an example, the final detection feature maps are 13 × 13, 26 × 26, and 52 × 52. Therefore, when using the clustering algorithm, the nine prior frames can be divided into three categories: small, medium, and large. The prior boxes are allocated according to the principle that small priori boxes correspond to large-size feature maps and large-size priori boxes correspond to small-size feature maps. The clustering algorithm used to obtain the prior frame size in YOLOv4 is the KMeans clustering algorithm. In this algorithm, the distance between the real frame size and the category center is different from the distance method adopted by the traditional clustering algorithm. The distance calculation method used in the clustering algorithm is the Euclidean distance, but when the size of the anchor boxes is large, it will introduce a large error. Therefore, it will use intersection-over-union (IoU) as the benchmark for distance judgment, and its distance function is shown as follows:

(1) $$\begin{array}{c} d_{\text{box},\text{centroid}}=1-{\text{IOU}}_{\text{box},\text{centroid}}. \end{array}$$

As shown in Figure 2, red represents the center of the cluster, that is, the anchor box is obtained by clustering; blue represents the real box; and the black part represents the overlapping part of the two, that is, the calculation of IOU is

(2) $$\begin{array}{c} {\text{IOU}}_{\text{box},\text{centroid}}=\frac{S_{\text{black}}}{S_{\text{red}}+S_{\text{blue}}-S_{\text{black}}}\\ =\frac{H⋆L}{H1*L1+H0*L0-H^{*}L}\;. \end{array}$$

After using the KMeans clustering algorithm to obtain the prior box, the three YOLO heads in the “Prediction” part in Figure 1 can be used for prediction. The sizes of the three YOLO heads are 13 × 13 × ((num_classes + 1 + 4) × 3), 26 × 26 × ((num_classes + 1 + 4) × 3), and 52 × 52 × ((num_classes + 1 + 4) × 3), where “num_classes” dimension information represents the prediction result of the classification and the category. The 1-dimensional information represents the confidence level of the predicted value, which indicates whether there is an object at the location. The 4-dimensional information represents the coordinate information of the predicted box, that is [*x*_offiset_, *y*_offset_, *h*, *w*], multiplied by 3, because each grid point on the feature layer has 3 a priori frames. We take the 13 × 13 YOLO head as an example. The 2-dimensional schematic diagram of the 13 × 13 feature map is shown in Figure 3. It can be expressed as dividing the picture into 13 × 13 grids, each grid is equipped with 3 clusters. Each priori box has classification information, confidence score, and coordinate information responsible for prediction. Assuming that the center of the detected object in a picture falls within the red area, the object is represented by the red in the red square and the upper left corner point is responsible for prediction. Assuming that the confidence score of the first anchor is the highest, the first anchor is adjusted according to the predicted result-$\left[\begin{array}{c} t_{x},t_{y},t_{w},t_{h} \end{array}\right]$.

Since the position information predicted by the network is processed by the sigmoid function, the *t*_*x*_, *t*_*y*_ value output by the network is normalized to between 0 and 1, and the coordinate information output by the network is the offset relative to the grid point, so the output information needs to be decoded accordingly. The decoding process can be shown in Figure 4, and the specific decoding calculation is shown in the following equations:

(3) $$\begin{array}{c} b_{x}=\sigma \left(t_{x}\right)+c_{x}, \end{array}$$

(4) $$\begin{array}{c} b_{y}=\sigma \left(t_{y}\right)+c_{y}, \end{array}$$

(5) $$\begin{array}{c} b_{w}=p_{w}e^{t_{w}}, \end{array}$$

(6) $$\begin{array}{c} b_{h}=p_{h}e^{t_{h}}, \end{array}$$

where the dotted line represents a priori box, *p*_*w*_ and *b*_*h*_ represent the width and height of the a priori box, and the blue box represents the result box obtained through network prediction and decoding, *σ* represents sigmoid activation function, and *c*_*x*_ and *c*_*y*_ represent the coordinates of the red grid points on the feature map. After the decoding of the above process, after the adjustment of the prior frame, the position information becomes the position information-[*b*_*x*_, *b*_*y*_, *b*_*w*_, *b*_*h*_].

After decoding the predicted results of the trained network, the target can be detected, and the category information and location information corresponding to the target can be obtained.

### 3.2. Improvement of YOLOv4

#### 3.2.1. Feature Fusion Improvement

In the basic YOLOv4 model, its feature fusion draws on the current mainstream fusion methods such as FPN [11], ASFF [12], PAN [13], BiFPN [14], and other fusion schemes. The fusion process is mainly in the “neck” part shown in Figure 1. The multiscale feature fusion process is shown in Figure 5.

As shown in Figure 5, the multiscale feature fusion process of YOLOv4 is mainly completed in the “neck” part. It not only uses the top-down structure in FPN but also uses the down-top structure. Since the semantic information between feature maps of different scales is different, the simple concatenation fusion method using FPN is not scientific, which results in the network not performing the fusion of information between high and low feature layers well. So after splicing, the YOLOv4 network uses the CBL structure to perform 5 common convolution operations and add learning coefficients on the basis of splicing, so that the network can perform adaptive feature fusion. The conventional feature fusion operation only uses the top-down structure. In YOLOv4, the down-top structure is superimposed on the top-down structure to make the feature fusion effect more effective.

Although feature fusion is fully carried out in YOLOv4, only the splicing operation is used in the process of feature map fusion, and this will ignore some of the associated information between the feature maps. For this reason, in this study, we modified the “Concat” and added the “Add” operation to make the fusion between feature maps more fully, the process is shown in Figure 6.

In each feature fusion process, a 5-layer CBL structure is used for convolution so that the model can better perform adaptive feature fusion. A total of four feature fusions are performed in the model, and the 5-layer CBL is run four times. The structure is shown in Figure 7.

#### 3.2.2. Attention Improvement

Affected by the SENet [15] and CBAM [16] models, in order to increase the model's attention to the target and remove some useless information, YOLOv4 uses a spatial attention mechanism after feature fusion. At the same time, in order to reduce the amount of calculation and balance the premise of the detection accuracy and detection speed, the spatial attention module (SAM) in CBMA is simply modified, and the spatial attention module is shown in Figure 8. In order to speed up the training of the network, this structure uses convolution operations instead of the original maximum pooling and mean pooling operations in the channel dimension and directly obtains the attention weight parameter. Because the input feature map and the attention information dimension are consistent, the two can be pointwise operated to get the output value.

YOLOv4 only uses the attention mechanism in the spatial dimension and only distributes the weight of the information in the space. But in the channel dimension, the information in each channel dimension represents a feature, but not all features play the same role. Some feature information in the channel dimension plays a small role or redundant information for detecting the target, while some feature information in the channel dimension plays a crucial role for target detection. After the feature fusion, the value in the channel dimension is multiplied, which brings more redundant information, so it is necessary to perform weight distribution in the channel dimension. Moreover, in the CBAM structure, it has been experimentally proved that the channel attention module (CAM) is often performed in front of the spatial attention so as to better play the role of attention. For this reason, the channel attention structure is designed in front of the spatial attention. The channel attention module is shown in Figure 9. The channel attention module in this study is modified on the basis of the channel attention module in CBAM. The channel attention in CBAM uses the maximum pooling and average pooling operations in the spatial dimension to compress the spatial dimension to 1, while retaining the channel dimension, and the two pooling results obtained are sent to a shared multi-layer perceptron for calculation. After accumulating the obtained results, the sigmoid activation function is used for processing so as to obtain the corresponding channel attention information. This research does not take the abovementioned form, but directly uses convolution to compress the spatial dimension, further improve the ability of attention learning, and finally obtain the weight distribution information on the corresponding channel.

The channel attention module is placed before the spatial attention module to form the attention module of this research. Its structure is shown in Figure 10. The weight distribution of the channel attention is performed first, and different feature maps are assigned. At the same time, on this basis, the weight distribution of spatial information is carried out in order to achieve the optimal effect.

### 3.3. Loss Function

The loss function used in this study is different from the commonly used target detection algorithm. In the box regression part, CIOU is used as the loss to optimize, and the calculation process is shown in the following equation:

(7) $$\begin{array}{c} \text{CIOU}=\text{IOU}-\frac{\rho^{2}\left(b,b^{gt}\right)}{c^{2}}-av. \end{array}$$

IOU represents the intersection ratio of the real box and the detection box, *ρ*^2^(*b*, *b*^*gt*^) represents the Euclidean distance between the center point of the real box and the detection box, *c* represents the diagonal distance of the smallest rectangular area that can include both the real box and the prediction box, and the calculation of the *a* and *v* are shown in the following equations:

(8) $$\begin{array}{c} a=\frac{v}{1-\text{IOU}+v}, \end{array}$$

(9) $$\begin{array}{c} v=\frac{4}{\pi^{2}}{\left(\arctan\frac{w^{gt}}{h^{gt}}-\arctan\frac{w}{h}\right)}^{2}. \end{array}$$

After the value of CIOU is obtained, the corresponding regression loss can be calculated. The calculation process is

(10) $$\begin{array}{c} {\text{LOSS}}_{\text{CIOU}}=1-\text{CIOU}\\ =1-\text{IOU}+\frac{\rho^{2}\left(b,b^{gt}\right)}{c^{2}}+av. \end{array}$$

The loss function used in the calculation of category loss and confidence loss is still the cross-entropy loss function, which is consistent with YOLOv3, and its calculation is

(11) $$\begin{array}{c} {\text{LOSS}}_{\text{conf}}=\sum_{i=0}^{K\times K}\sum_{j=0}^{M}I_{ij}^{\text{obj}}\left[{\hat{C}}_{i}\log\left(C_{i}\right)+\left(1-{\hat{C}}_{i}\right)\log\left(1-C_{i}\right)\right]\\ -\lambda_{\text{noobj}}\sum_{i=0}^{K\times K}\sum_{j=0}^{M}I_{ij}^{\text{noobj}}\left[{\hat{C}}_{i}\log\left(C_{i}\right)+\left(1-{\hat{C}}_{i}\right)\log\left(1-C_{i}\right)\right]\\ -\sum_{i=0}^{K\times K}I_{ij}^{\text{noobj}}\sum_{c\in \text{classes}}\left[{\hat{p}}_{i}\left(c\right)\log\left(p_{i}\left(c\right)\right)+\left(1-{\hat{p}}_{i}\left(c\right)\right)\log\left(1-p_{i}\left(c\right)\right)\right]. \end{array}$$

## 4. Experiment

### 4.1. Experiment Platform

The defect detection model in this research is a deep learning model that requires continuous iterative training. This process requires a lot of parallel computing. For this reason, it needs to be carried out on a computer with strong parallel computing capabilities. This research uses the deep learning workstation in the laboratory for training, and its main configuration information is shown in Table 1.

In terms of software systems, including operating systems, professional software, programming languages, deep learning frameworks, and corresponding auxiliary library files, the software system environment built in this study is shown in Table 2.

The specific hyperparameters are shown in Table 3.

In order to better train and converge the model, we use the idea of migration learning to initialize some parameters of the model's backbone network. This part mainly uses the model parameters trained on the ImageNet dataset to load into the backbone. In the network, the purpose of initialization is achieved. At the same time, the parameters of the rest of the model are initialized in a uniformly distributed manner, and the sample images of the training set are input into the network for forward propagation to obtain the prediction result. After decoding, the prediction results are compared with the real value, and the loss function of the model is calculated. The Adam algorithm is used to update the gradient of the loss function to realize the back propagation of the model. When the number of iterations of the model is set in advance, the training of the model is stopped. The model that can be tested is the same as the forward propagation process of the model training, but the NMS (nonmaximum suppression) needs to be executed later to further filter the output results of the network and finally get the model test results.

### 4.2. Experimental Result

In this experiment, three sets of experiments are compared for the surface defects of the two nonburr cylinder liners: raised and unsintered. There is basic YOLOv4, the detection model of the improved attention module, and the detection model of the improved attention and feature fusion. The three sets of experiments are performed on the same experimental platform and are consistent in terms of hyperparameter settings. The loss curve changes of the four model training processes are shown in Figure 11. It shows that the improved method can converge while training. The improvement in attention and the improvement of the feature fusion module converge faster than in the original model.

The above three models can basically converge after 300 epochs of iterative training. It is necessary to calculate and evaluate the corresponding evaluation indicators for the converged detection model. First, we calculate the precision and recall rate of each model accordingly. The classification precision curves and recall curves of the two categories under different thresholds in the basic model are shown in Figures 12 and 13. The classification precision curves and recall curves of each category of the attention improvement model at different thresholds are shown in Figures 14 and 15. Figures 16 and 17 show the classification precision and recall curves of each category of the model improved by the attention improvement and feature fusion modules at different thresholds at the same time.

It shows that it is hard to match models according to precision and recall rate curves. For the final evaluation, it is necessary to comprehensively consider the classification accuracy and recall rate to obtain the AP value and the final mAP value of each category for each model. The AP value calculation results are shown in Table 4, and the comparison results of mAP are shown in Figure 18.

Compared with the basic YOLOv4 model, the model improved by attention and feature fusion is improved. While the model is improving, the detection accuracy is also improving. As it can be seen in Figure 18, the improvement of the attention module brings a 1.5425% improvement to the model. Under the simultaneous action of the improved module of attention and the feature fusion module, the model has a 2.57% promotion.

After the test, the results of the detection speed of each model can be seen in Table 5. The improved model can realize real-time detection.

As it can be seen in Figure 19, the improved attention and feature fusion module are the best. Combining the previous evaluation indicators, we can know that the improvement of this research has an impact on detection accuracy. The promotion is effective.

## 5. Conclusion

This paper studies the deep learning-based surface defect detection technology of nonburr cylinder liners and proposes to improve the attention mechanism and feature fusion module based on YOLOv4. An experimental platform was built, and the training optimization method of the algorithm model was studied. Through three sets of experiments, the effects of different models were compared and evaluated. Experimental results show that our method has improved both accuracy and speed, and it can detect defects in production and realize industrialization. The algorithm mentioned in this paper has been verified by practical application with high accuracy and recognition efficiency, which can meet the needs of practical application. At the same time, how to implement online incremental learning of defect samples is the goal of the next research.

## Figures and Tables

**Figure 1:** YOLOv4 framework.

**Figure 2:** IOU diagram.

**Figure 3:** 13 × 13 size feature map division.

**Figure 4:** Predictive information decoding process.

**Figure 5:** Multiscale feature fusion process.

**Figure 6:** Improved feature fusion module.

**Figure 7:** 4 times 5xCBL structure.

**Figure 8:** Spatial attention module.

**Figure 9:** Channel attention module.

**Figure 10:** Improved attention module.

**Figure 11:** Loss function of each model.

**Figure 12:** Basic model precision curve.

**Figure 13:** Basic model recall curve.

**Figure 14:** Improved attention model precision curve.

**Figure 15:** Improved attention model recall curve.

**Figure 16:** Improved attention and feature fusion precision curve.

**Figure 17:** Improved attention and feature fusion recall curve.

**Figure 18:** MAP result of each model.

**Figure 19:** Comparison of test results of models.

**Table 1:** Hardware configuration information.

Hardware	Type/Num
CPU	Intel Core i7-7700 K/1
Motherboard	PRIME Z270-A/1
RAM	16G DDR4 2400 MHz/1
ROM	2TB/1
GPU	GeForce GTX 1080Ti/1

**Table 2:** Software system information.

Software	Type
Operating system	Ubuntu18.04
Programming platform	Pycharm community, Anaconda3
Programming language	Python3.7.0
Deep learning framework	PyTorch 1.4.0
others	NumPy, math, PTL, and pandas

**Table 3:** Model training hyperparameters.

Type	Data
Number of batches	8
Training times	300
Optimizer	Adam
Learning rate	1*e* − 3

**Table 4:** AP index comparison.

Detect Method	Input size	Raised	Unsintered
Basic model	416 × 416	97.66	88.49
Improved attention	416 × 416	98.52	89.59
Improved attention + feature fusion	416 × 416	98.63	89.96

**Table 5:** Detection speed comparison.

	Basic model	Improved attention	Improved attention + feature fusion
FPS	40.53	38.94	38.33

## Data Availability

No data were used to support this study.
